The article "Intratumoral Microbiota Impacts the First-Line Treatment Efficacy and Survival in Non-Small Cell Lung Cancer Patients Free of Lung Infection" was published in 2022. Journal: J Healthc Eng.

# Intratumoral Microbiota Impacts the First-Line Treatment Efficacy and Survival in Non-Small Cell Lung Cancer Patients Free of Lung Infection

**DOI:** 10.1155/2022/5466853

**Published:** 2022-02-07

**Authors:** Miao Zhang, Yan Zhang, Yi Sun, Shaochun Wang, Huan Liang, Yaguang Han

**Affiliations:** ^1^Department of Oncology, Graduate School, Hebei Medical University, Shijiazhuang 050017, China; ^2^Department of Oncology, Shijiazhuang People's Hospital, Shijiazhuang 050030, China

## Abstract

**Background:**

It has been known that there are microecology disorders during lung cancer development. Theoretically, intratumoral microbiota (ITM) can impact the lung cancer (LC) survival and treatment efficacy. This study conducted a follow-up investigation of non-small cell lung cancer (NSCLC) patients without lung infection to prove whether ITM indeed impacts the first-line treatment efficacy and survival.

**Methods:**

We enrolled all patients diagnosed with NSCLC in our department from 2017 to 2019, whose tumor samples were available (through surgery or biopsy) and sent for pathogen-targeted sequencing. All patients received the first-line treatment according to the individual situation. In the short term, the efficacy of the first-line treatment was recorded. During the follow-up, the survival status, progress events, and overall survival (OS) period were recorded if a patient was contacted.

**Results:**

Firstly, 53 patients were included, and our following analysis focused on the stage III and stage IV cases with ADC, SCC, or ASC tumors (47 cases). Several bacteria are associated with the LC status and progression, including N stages, metastasis sites, epidermal growth factor receptor (EGFR) mutation, first-line outcome, and later survival. The risk bacteria include *Serratia marcescens*, *Actinomyces neesii*, *Enterobacter cloacae*, and *Haemophilus parainfluenzae*; and the protective (against LC development and progression) ones include *Staphylococcus haemolyticus* and *Streptococcus crista*. In the logistic regression, the two-year survival can be predicted using the results of four bacteria (*Haemophilus parainfluenzae*, *Serratia marcescens*, *Acinetobacter jungii*, and *Streptococcus constellation*), with an accuracy rate of 90.7%.

**Conclusion:**

ITM have links to malignancy, EGFR mutation, first-line outcome, and survival of NSCLC. Our results implied the potential anti-NSCLC activity of antibiotics when used reasonably. It is still necessary to deepen the understanding of the characteristics of ITM and its interactions with NSCLC tumors and the immune cells, which is significant in individualized approaches to the LC treatment.

## 1. Introduction

Lung cancer (LC), especially non-small cell lung cancer (NSCLC), is one of the primary causes of global death. Traditionally, the carcinogenic factors of LC mainly include genetic factors and environmental factors. In recent years, it has been realized that microbial flora possibly impacts LC development [1]. The role of the microbiome has become increasingly clear, and variation of the microecology has been noticed in LC patients [2]; different clinicopathologies may be related to different conditions of the lung microbiota (LM) [3]. LM is also involved in LC onset and malignant progression. Understanding the diverse contributions of the bacterial microbiota to carcinogenesis is of great importance in LC diagnosis and treatment. Currently, studies do not distinguish LC cases with or without lung infection (LI). Bacterial and viral infections had influence on the patients' prognosis, affecting the immune system and impairing the outcome of anticancer treatments [4]. These cases have two major diseases, and the situation should be more complicated than LC alone. For patients free of LI, the features of tumor-associated microbiota are particularly informative in the investigation of tumorigenesis driven by LM. Additionally, published studies concerning the intratumoral microbiota (ITM) mainly focused on the basal clinical characteristics. Theoretically, IMT may impact the immune response and inhibit the treatment efficacy. So far, these factors and consequences are poorly understood in LC. It is reasonable to evaluate whether these interactions can impact the LC survival and treatment efficacy. However, very limited studies have analyzed the prognosis and investigated these potential influences induced by ITM.

The article "Intratumoral Microbiota Impacts the First-Line Treatment Efficacy and Survival in Non-Small Cell Lung Cancer Patients Free of Lung Infection" was published in 2022. Journal: J Healthc Eng.

Here, we conducted this 5-year follow-up study of NSCLC patients without respiratory infection and proved that ITM indeed impacts the first-line treatment efficacy and survival, which will show the potential anti-NSCLC activity of antibiotics. It is still necessary to deepen the understanding of the characteristics of ITM and its interactions with NSCLC tumors and the immune cells, which is significant in individualized approaches to the LC treatment.

## 2. Materials and Methods

### 2.1. Patients

We enrolled all patients diagnosed NSCLC in our department since 2017, whose tumor samples were available (through surgery or biopsy) and sent for pathogen-targeted sequencing. The inclusion criteria are as follows: (1) patients diagnosed with lung cancer, including adenocarcinoma (ADC), squamous cell carcinoma (SCC), and adenosquamous carcinoma (ASC) and (2) patients with the basic demographic information and tumor characteristics. The exclusion criteria are as follows: (1) patients diagnosed with a definite respiratory infection and other system disease. The smoking history and average number of cigarettes smoked every year were acquired. The EGFR and TP53 mutation features were extracted from the electronic medical record system. In addition, 5 *μ*m paraffin-embedded tumor-tissue sections were prepared, and the PD-L1 expression in the immunohistochemistry analysis was acquired from the Department of Pathology. All patients received the first-line treatment according to an individual situation. In the short term, the efficacy of the first-line treatment was recorded. During the follow-up (at most 5 years), the survival status, progress events, progression-free survival (PFS), and overall survival (OS) period were recorded if a patient was contacted.

The article "Intratumoral Microbiota Impacts the First-Line Treatment Efficacy and Survival in Non-Small Cell Lung Cancer Patients Free of Lung Infection" was published in 2022. Journal: J Healthc Eng.

### 2.2. Targeted Sequencing of Intratumoral Microbiota (ITM)

We used all the collected tumor samples to perform the pathogen-targeted sequencing. The sequencing process was performed in the Pathogeno One Pan-Infectious Pathogen high-throughput sequencing system by Shanghai Bingyuan Medical Technology Co. The report of each patient was acquired and documented in the dataset. For each known pathogenic microorganism, two fields were used for analysis: the reads of known bacteria and the presence of each microorganism.

### 2.3. Outcome Measures

53 patients were included, and 47 cases were followed for analysis.

The risk bacteria include *Serratia marcescens*, *Actinomyces neesii*, *Enterobacter cloacae*, and *Haemophilus parainfluenzae*; the protective (against LC development and progression) ones include *Staphylococcus haemolyticus* and *Streptococcus crista*.

### 2.4. Statistical Analysis

The data are expressed as numbers with proportions (%), mean with SD, or median with 95% confidence interval (CI). The differences in values derived from categorical variables were compared using the chi-squared test. One-way ANOVA was used for three or four groups. Overall survival (OS) in relation to the bacterial result was evaluated by Kaplan–Meier survival curve and log-rank test. The Cox proportional hazard model was also used to discover the potential risk of the relationship between multiple factors and the overall postoperative survival. Statistically significant prognostic factors identified by univariate analysis were further included in the multivariate analysis. A *P* value <0.05 was considered statistically significant.

## 3. Results

### 3.1. Clinical Characteristics of Enrolled NSCLC Patients

Firstly, 53 patients were included, and the clinical features are presented in Table 1. There were 38 (71.7%) males and 15 (28.3%) females. About 40% of patients were smokers. There were 25 (47.2%) stage III and 25 (47.2%) stage IV cases. Only three patients were in stage I or II. The pathological types were as follows: the numbers for adenocarcinoma (ADC), squamous cell carcinoma (SCC), and adenosquamous carcinoma (ASC) were 26 (49.1%), 21 (39.6%), and 3 (5.7%), respectively. Besides, there were three cases of other types, including two poorly differentiated carcinomas and one large cell lung cancer. The main metastasis sites were mediastinal lymph nodes, lung, bone, liver, and brain.

The article "Intratumoral Microbiota Impacts the First-Line Treatment Efficacy and Survival in Non-Small Cell Lung Cancer Patients Free of Lung Infection" was published in 2022. Journal: J Healthc Eng.

### 3.2. Association between Intratumoral Microbiota (ITM) and Disease Characteristics

Given there were only three stage-I/II cases, and only three cases had the other pathological types (including poorly differentiated carcinoma and large cell lung cancer), our following analysis focused on the stage III and stage IV cases with ADC, SCC, or ASC tumors (47 cases). If some microbiota had no more than four positive cases, the results might be unreliable. Therefore, those microbiota results with rare cases were culled from the raw data. First, the association between the microbiota and the pathological type was probed. Among ADC, SCC, and ASC, the ASC tumors had a higher abundance of *Serratia marcescens* (2.67 ± 4.619 counts) versus ADC (0.27 ± 0.962 counts, *P* < 0.05) and SCC (0 counts, *P* < 0.05). However, the case number of ASC was three, and this conclusion is still to be verified. Next, there was no association between ITM and the major stage (T stage and M stage). But for N stages, among N0 to N3, we noticed different features in the presence of *Actinomyces neesii* and *Haemophilus* (Table 2). These two bacteria were negatively related to the metastasis in the lymph node (*P* < 0.01). Next, the main metastasis organs/tissues (including mediastinal lymph nodes, lung, bone, liver, brain, and pleura) showed noticeable association with the ITM. Tumors with *Serratia marcescens* were more likely to develop brain metastasis (*P* < 0.01, Table 3), and those with *Enterobacter cloacae* were more likely to develop metastases to the mediastinal lymph node (*P* < 0.05, Table 3). Moreover, for the first time, we noticed that ITM can link to the EGFR mutation (Table 4). For example, EGFR mutation was negatively related to *Haemophilus parainfluenzae* (*P* < 0.05) but positively with *Serratia marcescens* (*P* < 0.01). Furthermore, *Acinetobacter jungii* was positively correlated with PD-L1 expression (PD-L1 positive/negative = 4/8) in *Acinetobacter jungii*-positive cases, in comparison with 7/41 in *Acinetobacter jungii*-negative cases, (chi-square = 4.168, *P* = 0.041). Collectively, ITM is notably associated with disease characteristics of NSCLC.

The article "Intratumoral Microbiota Impacts the First-Line Treatment Efficacy and Survival in Non-Small Cell Lung Cancer Patients Free of Lung Infection" was published in 2022. Journal: J Healthc Eng.

### 3.3. Association between ITM and the First-Line Treatment Outcomes

Next, we evaluated whether ITM may impact the efficacy of first-line treatments (targeted therapy or chemotherapy). Also, only stage III and IV cases were analyzed. Overall, there is no association between ITM and the response to the first-line treatment. However, in the hierarchical analysis, we noticed that the presence of *Haemophilus parainfluenzae* was negatively correlated with response to the first-line treatment for stage IV patients (Table 5). The patients with intratumoral *Haemophilus parainfluenzae* had a poorer control rate (3/6 vs 18/19).

### 3.4. Association between ITM and Survival

Initially, we used the Kaplan–Meier method to evaluate the association between ITM and survival in stages III and IV. If any case, the number of the ITM/target event (progressed or death) double-positive set was not more than two, this index was omitted. Similar to the response to the first-line treatment outcomes, the presence of *Haemophilus parainfluenzae* was related to the poorer PFS of stage IV patients (Table 6 and Figure 1(a)). When stage III and IV cases were pooled together, we found that *Staphylococcus haemolyticus* infection was linked to the longer PFS (Table 7 and Figure 1(b)). Meanwhile, for pooled cases (stage III and IV), *Serratia marcescens* was related to better OS (Table 8 and Figure 1(c)) and the presence of *Haemophilus parainfluenzae* was related to the poorer OS (Table 9 and Figure 1(d)). Also, the Cox regression analysis (using the Enter model) showed that, besides *Staphylococcus haemolyticus*, *Streptococcus crista* is also associated with better PFS (Table 10). On the contrary, *Haemophilus parainfluenzae* and *Corynebacterium jergeri* were two risk factors for OS (Table 11). Finally, in the logistic regression model, the two-year survival was predicted (for stage III or IV patients with ADC, SCC, or ASC), using the following seven variables: age, major stage, pathological type, and the results of four bacteria (*Haemophilus parainfluenzae*, *Serratia marcescens*, *Acinetobacter jungii*, and *Streptococcus constellation*). The variables and their contribution are listed in Table 12. Using this regression, the predicted results (at the cutoff value 0.5) are as follows: 31 true-negative cases, 1 false-positive case, 3 false-negative cases, and 8 true-positive cases (with an accuracy rate of 90.7%).

## 4. Discussion

It has been recognized that LC has non-negligible links to pathogenic microorganisms, such as *Haemophilus influenzae*, *Moraxella catarrhalis*, *Granulicatella*, *Abiotrophia*, *Streptococcus*, and *Mycobacterium tuberculosis* [5–8]. With the development of sequencing technology, their relationships have been increasingly clear. However, there are still problems to be solved. One of the most important questions is whether and how ITM affect the treatment and prognosis of lung cancer. We here innovatively observed the link between ITM and disease characteristics and combined the results of ITM to construct a prognostic model. Overall, several bacteria are associated with the LC status and progression, including N stages, metastasis sites, EGFR mutation, first-line outcome, and later survival. Seemingly, the risk bacteria include *Serratia marcescens*, *Actinomyces neesii*, *Enterobacter cloacae*, and *Haemophilus parainfluenzae*; and the protective (against LC development and progression) ones include *Staphylococcus haemolyticus* and *Streptococcus crista*. So far, all the abovementioned associations were highly novel findings, so supporting evidence are limited. *Haemophilus parainfluenzae* has been regarded as an indicator of LM changes triggered by preoperative prophylaxis in LC patients [9]. It was observed in 43.3% to 63.3% cases of LC patients [9], and it is reasonable to believe that this bacterium is a cancer-promoting strain. Interestingly, there are also some seemingly unsupportive evidence. For example, prodigiosin is a secondary metabolite, isolated from a culture of *Serratia marcescens*. It induces LC apoptosis in both caspase-dependent and caspase-independent pathways [10]. It is still early to tell whether *Serratia marcescens* has a driving or suppressive effect on LC. However, based on Table 3, if *Serratia marcescens* drives LC progression, a possible pathway is metastasis in the brain. Similarly, as shown in Table 2, the reason for the driving effect by *Actinomyces neesii* may be due to the promotion of lymph node metastasis. Also, *Haemophilus parainfluenzae*, as a risk factor to survival, may promote the EGFR-WT carcinomas but not EGFR mutant ones, and these cases cannot be treated by targeted TKIs, which is a possible reason for the poor survival.

The article "Intratumoral Microbiota Impacts the First-Line Treatment Efficacy and Survival in Non-Small Cell Lung Cancer Patients Free of Lung Infection" was published in 2022. Journal: J Healthc Eng.

The mechanisms underlying the impact of ITM on survival may include the following and various aspects. First, ITM (as well as bacteria outside the tumor) may drive carcinogenesis directly. It is estimated that 20% of cancers are caused by infectious agents [11]. The dysbiosis of some carcinogenic microbiomes causes direct DNA damage and inflammation [12]. Moreover, inflammation triggered by microbial dysregulation can largely impact invasion and angiogenesis, which significantly drives the malignant progression. Known targets of microbiome-induced inflammation include TLRs, NF-ĸB, and STAT3 [13–15]. These direct effects exerted by microbes are highly possibly carcinogenic. Also, there are some indirect mechanisms. For example, through modulation of immune response, the response to treatment and prognosis can be influenced. Besides, the inflammatory effect triggered by IMTs, their inhibitive effects on the immune system can also play an essential role [12]. At least partially, ITM can result in the exhaustion of immune cells, and they inhibit antitumor immunity together with the tumor cells. For example, they may exert suppress NK cells [16]. However, given the digestive tract has more abundant flora, most attention to the relationship between microbiome and cancer has been paid to colorectal cancer and gastric cancer. There are limited data about the impact of ITM on the prognosis of LC, but related research can be used as reference. Recently, a Chinese study found nine enriched bacteria in the lung of NSCLC patients [17]. Also, the analysis of T cells and B cells implied that these bacteria in the lung may change the immune cell infiltration in LC tissues. Recently, a retrospective study of 69 NSCLC reported that patients treated with anti-PD-1 antibodies receiving antibiotics had greatly decreased objective response rate, OS, and PFS compared to those who did not use antibiotics [18]. This result highlights that inappropriate usage of antibiotics may influence the flora of the tumor environment and impair the treatment effect. Indeed, the use of antibiotics has been reported to be associated with an elevated risk of LC onset [19, 20]. Moreover, when not limited to the local lung tissue, another interesting issue is whether the gut-lung axis may impact the outcome of chemotherapy and later survival through the impact of microbiota. This issue is being investigated by a multicenter, prospective, double-blind randomized trial [21], but the final result has not yet been announced.

Still, the present study has some limitations. The main shortcoming is the small sample size. The number of many classification results was around 5 in one cell, which is the major reason for the inconsistency between the univariate analysis and binary regression analysis. Also, due to the limited sample size, the performance of bacteria in the 2-year prediction model is not outstanding enough, and we cannot divide the dataset into the training set and test set; hence, the scalability of the model is still unclear.

## 5. Conclusion

This novel study proved that ITM was related to malignancy, EGFR mutation, first-line outcome, and survival of NSCLC. Also, our results implied the potential anti-NSCLC activity of antibiotics when used reasonably. It is still necessary to deepen the understanding of the characteristics of ITM and its interactions with NSCLC tumors and the immune cells, which is significant in individualized approaches to the LC treatment.

The article "Intratumoral Microbiota Impacts the First-Line Treatment Efficacy and Survival in Non-Small Cell Lung Cancer Patients Free of Lung Infection" was published in 2022. Journal: J Healthc Eng.

## Figures and Tables

**Figure 1:** The association between intratumoral microbiota and survival in stage III and IV non-small cell lung cancer patients using the Kaplan–Meier method. (a) The presence of *Haemophilus parainfluenzae* was related to poorer PFS (only for stage IV patients). (b) *Staphylococcus haemolyticus* infection was linked to longer progression-free survival (PFS). (c) *Serratia marcescens* was related to better overall survival (OS). (d) *Haemophilus parainfluenzae* was related to poorer OS.

**Table 1:** Clinical characteristics of NSCLC patients.

Characteristics		Case number	%
Total cases		53	100
Gender	Male	38	71.7
	Female	15	28.3

Smoking history	Never smoking	21	39.6
	Smoking	31	58.5
	Smoking quitted	1	1.9

Major stage	I	1	1.9
	II	2	3.8
	III	25	47.2
	IV	25	47.2

Pathological type	ADC	26	49.1
	SCC	21	39.6
	ASC	3	5.7
	Others	3	5.7

PD-L1 positive		13	24.5
EGFR mutation		12	22.6
Metastasis	Mediastinal lymph nodes	11	20.8
	Lung	11	20.8
	Bone	10	18.9
	Liver	7	13.2
	Brain	6	11.3
	Pleura	3	5.7

	N	Mean	SD
Age (years)	53	66.08	8.786
Cigarettes per year	53	385.85	436.813

**Table 2:** Association between ITM and N stages.

Bacteria		N0	N1	N2	N3	Chi-square	*P* value
*Actinomyces neesii*	−	0	1	28	8	18.875	<0.001
	+	1	1	1	0		

*Haemophilus*	−	0	2	25	8	8.473	0.037
	+	1	0	4	0		

**Table 3:** Association between ITM and metastasis sites.

Bacteria		No	Yes	Chi-square	*P* value
Brain					
*Serratia marcescens*	−	39	4	8.136	0.004
	+	1	2		

Mediastinal lymph node					
*Enterobacter cloacae*	−	36	6	6.031	0.014
	+	2	3		

**Table 4:** Association between ITM and EGFR mutation.

Bacteria		WT	Mutant	Chi-square	*P* value
*Haemophilus parainfluenzae*	−	24	12	4.924	0.026
	+	11	0		

*Serratia marcescens*	−	34	9	9.093	0.003
	+	0	3		

**Table 5:** Association between *Haemophilus parainfluenzae* and the first-line outcome in stage IV.

Bacteria		PD	SD	PR	Chi-square	*P* value
*Haemophilus parainfluenzae*	−	1	10	8	6.877	0.032
	+	3	2	1		

**Table 6:** Association between *Haemophilus parainfluenzae* and the PFS in stage IV.

Outcome	Median	95% CI		Log-rank chi-square	*P* value
−	7 months	4.891	9.109	3.940	0.047
+	4 months	1.600	6.400		

**Table 7:** Association between *Staphylococcus haemolyticus* and the PFS.

Outcome	Median	95% CI		Log-rank chi-square	*P* value
−	7 months	6.102	7.898	5.887	0.015
+	Not reached				

**Table 8:** Association between *Serratia marcescens* and the OS.

Outcome	Median	95% CI		Log-rank chi-square	*P* value
−	18 months	15.107	20.893	6.995	0.008
+	49	N.A.	N.A.		

The article "Intratumoral Microbiota Impacts the First-Line Treatment Efficacy and Survival in Non-Small Cell Lung Cancer Patients Free of Lung Infection" was published in 2022. Journal: J Healthc Eng.

**Table 9:** Association between *Haemophilus parainfluenzae* and the OS.

Outcome	Median	95% CI		Log-rank chi-square	*P* value
−	20 months	18.676	21.324	4.933	0.026
+	14 months	5.368	22.632		

**Table 10:** Cox regression analysis of PFS based on IMT results.

Bacteria	B	Wald	*P* value	Exp (B)
*Enterococcus*	−0.199	0.131	0.717	0.820
*Streptococcus crista*	−1.216	3.951	0.047^*∗*^	0.297
*Acinetobacter jungii*	0.380	0.379	0.538	1.462
*Aerococcus* light green	0.115	0.041	0.840	1.121
*Staphylococcus haemolyticus*	−2.588	5.715	0.017^*∗*^	0.075
*Haemophilus haemolyticus*	0.267	0.209	0.648	1.306
*Actinomyces neesii*	0.643	0.696	0.404	1.901
*Corynebacterium pseudodiphtheriae*	0.468	0.614	0.433	1.596
*Streptococcus constellation*	0.217	0.091	0.762	1.242
*Streptococcus pneumoniae*	0.102	0.048	0.827	1.107
*Haemophilus parainfluenzae*	0.966	2.681	0.102	2.627
*Prevotella* II	0.460	0.497	0.481	1.584
*Haemophilus influenzae*	0.463	0.502	0.479	1.589
*Haemophilu*s	0.018	0.001	0.978	1.018
*Corynebacterium jergeri*	0.450	0.612	0.434	1.569
*Enterobacter cloacae*	−1.070	2.556	0.110	0.343
*Serratia marcescens*	−0.881	1.410	0.235	0.415

**Table 11:** Cox regression analysis of OS based on IMT results.

Bacteria	B	Wald	*P* value	Exp (B)
*Enterococcus*	0.161	0.079	0.778	1.175
*Streptococcus crista*	−1.592	4.151	0.042^*∗*^	0.203
*Acinetobacter jungii*	0.042	0.005	0.946	1.043
*Aerococcus* light green	−0.670	0.962	0.327	0.512
*Staphylococcus haemolyticus*	−13.925	0.002	0.964	0.000
*Haemophilus haemolyticus*	0.974	2.297	0.130	2.649
*Actinomyces neesii*	−0.725	0.741	0.389	0.484
*Corynebacterium pseudodiphtheriae*	0.973	1.644	0.200	2.646
*Streptococcus constellation*	−0.776	0.816	0.366	0.460
*Streptococcus pneumoniae*	−0.777	1.980	0.159	0.460
*Haemophilus parainfluenzae*	1.396	4.771	0.029^*∗*^	4.038
*Prevotella* II	0.092	0.015	0.904	1.096
*Haemophilus influenzae*	−0.527	0.377	0.539	0.590
*Haemophilus*	0.278	0.130	0.718	1.320
*Corynebacterium jergeri*	1.997	6.086	0.014^*∗*^	7.366
*Enterobacter cloacae*	−0.799	1.629	0.202	0.450
*Serratia marcescens*	−13.556	0.003	0.960	0.000

**Table 12:** Logistic regression analysis of 2-year survival based on general information and IMT results.

Variables	B	Wald	*P* value	Exp (B)
Age	−0.189	2.512	0.113	0.827
Major stage	−1.118	0.513	0.474	0.327
Pathological type		0.000	1.000	
ADC	−21.501	0.000	0.998	0.000
SCC	−19.736	0.000	0.999	0.000
ASC	−20.288	0.000	0.999	0.000
*Haemophilus parainfluenzae*	−0.049	0.001	0.974	0.952
*Serratia marcescens*	41.742	0.000	0.999	1.3^*∗*^10^∧^18
*Acinetobacter jungii*	0.336	0.029	0.864	2.1^*∗*^10^∧^9
*Streptococcus constellation*	19.164	0.000	0.998	2.1^*∗*^10^∧^8

## Data Availability

The data used to support this study are available from the corresponding author upon request.
